The article "Modeling the Dynamics of Coronavirus Disease Pandemic Coupled with Fear Epidemics" was published in 2021. Journal: Comput Math Methods Med.

# Modeling the Dynamics of Coronavirus Disease Pandemic Coupled with Fear Epidemics

**DOI:** 10.1155/2021/6647425

**Published:** 2021-03-11

**Authors:** Saul C. Mpeshe, Nkuba Nyerere

**Affiliations:** ^1^Department of Mathematical Sciences, University of Iringa, P.O. Box 200, Iringa, Tanzania; ^2^Department Mathematics, Informatics and Computational Science, Sokoine University of Agriculture, P.O. Box 3000, Morogoro, Tanzania

## Abstract

A modeling approach to investigate the dynamics of COVID-19 epidemics coupled with fear is presented in this paper. The basic reproduction number *R*_0_ is computed and employed in analysing the effect of initial transmission and the conditions for disease control or eradication. Numerical simulations show that whenever there is an outbreak coupled with fear, the disease is likely to persist in the first two months, and after that, it will start to slow down as the recovery rate from fear increases. An increase in the number of recovered individuals lead to a rise in the number of susceptibles and consequently set off a second wave of infection in the third month of the epidemic.

## 1. Introduction

### 1.1. Coronavirus Disease Outbreak

According to the World Health Organisation (WHO), coronavirus disease (COVID-19) is a disease caused by a new coronavirus called SARS-CoV-2. WHO first learned of this new virus on December 31st, 2019, following a report of a cluster of cases of ‘viral pneumonia' in Wuhan, People's Republic of China [1].

The COVID-19 virus spreads primarily through droplets of saliva or discharge from the nose when an infected person coughs or sneezes. Most people infected with the COVID-19 virus will experience mild to moderate respiratory illness and recover without requiring special treatment. Older people and those with underlying medical problems like cardiovascular disease, diabetes, chronic respiratory disease, and cancer are more likely to develop severe illness [2].

Since its outbreak in December 2019, COVID-19 has caused a great threat worldwide, with millions of people being infected and dying. By November 30th, 2020, cases of coronavirus were about 63 millions, with death cases of about 1.5 million and recovery cases of about 43.5 millions [3].

The COVID-19 pandemic has attracted researchers in different fields, including mathematics, to analyse, predict, and give suggestions on the disease outbreak's dynamics and how to control it. Since the outbreak of COVID-19, different mathematical models for the dynamics of COVID-19 have been developed. Approaches used include simple compartmental models, network models, age-structured models, discrete models, and stochastic models. Ndairou et al. [4] developed a compartmental mathematical model that has taken into account the superspreading phenomenon of individuals. In this model, the basic reproduction number was computed, and the sensitivity of each parameter value was analysed. The stability of the disease-free equilibrium was also analysed.

Liu et al. [5] developed an SEIRU mathematical model to study the latency period's impact with a constant time delay. Wang et al. [6] developed an SEIR, which was applied to estimate the epidemic trend in Wuhan, China. A simple susceptible infected-recovered-deaths (SIRD) model, which uses an indicative rate of recovery based on the kinetic parameter, was also developed by Fanelli and Piazza [7].

A stochastic susceptible, exposed, infectious, treated, and recovered (SEITR) model with input options for multiple stages of infection, treatment, and the external fluctuations in the transmission were developed by Otunuga and Ogunsolu [8]. Jayson et al. [9] developed a spatiotemporal “risk source” model with an index for assessing transmission risk that leverages population flow data over time for different locations. The changes in distribution and growth of epidemic overtime were derived using a Cox proportional hazards framework with a time-varying hazard rate function that describes the number of cumulative confirmed cases at any given time for a given population.

A discrete-time SIR model with dead individuals, based on the official counts for confirmed cases, was developed by Anastassopoulou et al. [10]. The model was a data-based model aimed at analysing and forecasting the COVID-19 outbreak.

Casella [11] developed a control-oriented SEIR model that stresses the effects of delays and compares the outcome of different containment policies. The goal, in this case, was to reduce the reproduction number and control the epidemic. Other models with control measures include that of Mumbu and Hugo [12], Cakan [13], Vega [14], the SIDARTHE model by Giulia et al. [15], and the SEIRQ epidemic model by Hu et al. [16].

Mathematical models that use fractional derivatives have also been formulated. Alkahtani and Alzaid [17] developed a novel mathematical model of COVID-19 with fractional derivative in which the basic reproduction number and stability were analysed. Tuan et al. [18] formulated a mathematical model of COVID-19 using Caputo fractional derivative. Other COVID-19 models formulated using fractional derivatives includes Khan et al. [19], Awais et al. [20], and Khan and Atangana [21].

### 1.2. Coupling Fear in Epidemics

Outbreaks of any infectious disease can be associated with fear to society, especially when the disease causes severe illness and death. Fear, if not controlled, can do more damage than a disease virus can do. Controlling fear among infected and noninfected individuals can be an important aspect in controlling disease transmission. While fear is an emotion that we frequently experience as an individual, it can also be a shared and social emotion, which circulate through groups and communities, and shapes our reaction to ongoing events. Like other emotions, fear is contagious and can spread swiftly [22]. Fear may also cause individuals to isolate themselves as a reaction to the epidemic crisis. People may isolate on an individual basis, or a household basis [23].

Though fear is contagious, hardly few models have incorporated its impacts. Epstain et al. [24] developed a mathematical and computational model coupled with contagion disease and fear dynamics and found that fear has a great impact on disease transmission and control. Valle et al. [23] developed a model on the impact of behaviour changes on the spread of pandemic influenza in which fear-based home isolation was considered one of the behaviour changes.

Fear has played a significant role in the coverage of the coronavirus outbreak. There have been a prominence of anxiety as a theme in reports of the coronavirus which support that much of the scope of the epidemic is more a reflection of public fear than information of what is happening in terms of the spread of the virus [22].

In this article, we develop a mathematical model using nonlinear differential equations. Our model captures the dynamics of COVID-19 infection coupled with the fear epidemics. To gain some insights into disease vital dynamics, we establish the basic reproduction number which is the initial transmission of the disease, determine the existence and stability of equilibrium points, and analyse the impact of fear on the dynamics of COVID-2019. Over time, mathematical models have been used to describe the transmission dynamics of several infectious diseases as well as the possible control mechanisms available for the disease [25].

## 2. The COVID-19 Model Coupled with Fear

### 2.1. Model Formulation

The model considers only human population with natural death rate, disease-induced death rate, and the fear-induced death rate for human. The population consists of susceptible human (*S*), human infected with COVID-19 virus only (*I*_*c*_), human infected with both COVID-19 virus and fear (*I*_*cf*_), human with fear of contagion (*I*_*f*_), and recovered human (*R*).

It is assumed that individuals affected by fear will tend to go for self-isolation on their free will to form a compartment (*I*_*f*_). Meanwhile, individuals affected by the COVID-19 virus or both COVID-19 virus and fear will go for self-isolation or hospitalization compartment (*I*_*cf*_). The human with fear of contagion may recover from fear and become fearless susceptible. It is also assumed that an individual can develop fear from *I*_*c*_, *I*_*cf*_, and *I*_*f*_ but may contract disease only by contact with *I*_*c*_ and *I*_*cf*_ or infected objects.

Lockdown and other preventive measures such as social distancing and sanitization are not considered in this model.  Table 1 shows the model parameters and their description as they have been used in this work. As a framework to the approach used in this work, we mention the work by Epstain et al. [24] and Valle et al. [23].

Figure 1 shows the transmission dynamics of coronavirus fever with variables and parameters as described in Table 1. Using the parameters in Table 1 and Figure 1, an SISR model is derived using first-order nonlinear ordinary differential equations as follows:

(1) $$\begin{array}{c} \frac{dS}{dt}=\Lambda -\left(1-\alpha \right)\beta S\left(I_{c}+I_{cf}\right)-\left(1-\beta \right)\alpha S\left(I_{f}+I_{c}+I_{cf}\right)-\alpha \beta S\left(I_{c}+I_{cf}\right)-d_{n}S+\omega I_{f},\\ \frac{dI_{c}}{dt}=\left(1-\alpha \right)\beta S\left(I_{c}+I_{cf}\right)-\alpha I_{c}\left(I_{cf}+I_{f}\right)-\left(d_{n}+d_{c}+\gamma_{c}\right)I_{c},\\ \frac{dI_{cf}}{dt}=\alpha \beta S\left(I_{c}+I_{cf}\right)+\beta I_{f}\left(I_{cf}+I_{c}\right)+\alpha I_{c}\left(I_{cf}+I_{f}\right)-\left(d_{n}+d_{cf}+\gamma_{cf}\right)I_{cf},\\ \frac{dI_{f}}{dt}=\left(1-\beta \right)\alpha S\left(I_{f}+I_{c}+I_{cf}\right)-\beta I_{f}\left(I_{cf}+I_{c}\right)-\left(\omega +d_{n}+d_{f}\right)I_{f},\\ \frac{dR}{dt}=\gamma_{c}I_{c}+\gamma_{cf}I_{cf}-d_{n}R. \end{array}$$

### 2.2. Feasibility of the Model Solution

From the model equation, we have

(2) $$\begin{array}{c} \frac{dN}{dt}=\frac{dS}{dt}+\frac{dI_{c}}{dt}+\cdots +\frac{dR}{dt}\leq \Lambda -d_{n}N. \end{array}$$

Solving this equation, we obtain

(3) $$\begin{array}{c} 0\leq N\left(t\right)\leq \frac{\Lambda }{d_{n}}+N\left(0\right)\exp^{-d_{n}t}. \end{array}$$

As *t*⟶0, we have 0 < *N*(*t*) ≤ *Λ*/*d*_*n*_. Hence, the model solution is feasible and positively invariant in the region

(4) $$\begin{array}{c} \Omega =\left\{\left(S,I_{c},I_{cf},I_{f},R\right)\geq 0\in {\mathbb{R}}_{+}^{5}:S+I_{c}+I_{cf}+I_{f}+R\leq \frac{\Lambda }{d_{n}}\right\}. \end{array}$$

Since *R* does not appear in other equations, then the equation for *R* can be omitted from the analysis for its value can be obtained when the values for *S*, *I*_*c*_,  *I*_*cf*_, and *I*_*f*_ are known. The remaining system becomes

(5) $$\begin{array}{c} \frac{dS}{dt}=\Lambda -\left(1-\alpha \right)\beta S\left(I_{c}+I_{cf}\right)-\left(1-\beta \right)\alpha S\left(I_{f}+I_{c}+I_{cf}\right)-\alpha \beta S\left(I_{c}+I_{cf}\right)-d_{n}S+\omega I_{f},\\ \frac{dI_{c}}{dt}=\left(1-\alpha \right)\beta S\left(I_{c}+I_{cf}\right)-\alpha I_{c}\left(I_{cf}+I_{f}\right)-\left(d_{n}+d_{c}+\gamma_{c}\right)I_{c},\\ \frac{dI_{cf}}{dt}=\alpha \beta S\left(I_{c}+I_{cf}\right)+\beta I_{f}\left({\text{I}}_{cf}+I_{c}\right)+\alpha I_{c}\left(I_{cf}+I_{f}\right)-\left(d_{n}+d_{cf}+\gamma_{cf}\right)I_{cf},\\ \frac{dI_{f}}{dt}=\left(1-\beta \right)\alpha S\left(I_{f}+I_{c}+I_{cf}\right)-\beta I_{f}\left(I_{cf}+I_{c}\right)-\left(\omega +d_{n}+d_{f}\right)I_{f}. \end{array}$$

Thus, the model solution is feasible and positively invariant in the region

(6) $$\begin{array}{c} \Omega =\left\{\left(S,I_{c},I_{cf},I_{f}\right)\geq 0\in {\mathbb{R}}_{+}^{4}:S+I_{c}+I_{cf}+I_{f}\leq \frac{\Lambda }{d_{n}}\right\}. \end{array}$$

The existence of the feasible solution of the model, which is positively invariant in ℝ_+_^4^, implies that the model system is well-posed epidemiologically and mathematically. The well-posedness of the model allows us to continue with other mathematical treatments of the model.

### 2.3. Equilibrium Points

Setting the LHS of the model equation equal to zero and that *I*_*c*_ = *I*_*cf*_ = *I*_*f*_ = 0, we have the disease-free equilibrium *E*_0_ given by

(7) $$\begin{array}{c} E_{0}=\left(\frac{\Lambda }{d_{n}},0,0,0\right). \end{array}$$

The endemic equilibrium is *E*^∗^ = (*S*^∗^, *I*_*c*_^∗^, *I*_*cf*_^∗^, *I*_*f*_^∗^), where

(8) $$\begin{array}{c} S^{*}=\frac{1}{d_{n}}\left[\Lambda -\left(d_{n}+d_{c}+\gamma_{c}\right)I_{c}^{*}+\left(d_{n}+d_{cf}+\gamma_{cf}\right)I_{cf}^{*}+\left(d_{n}+d_{f}\right)I_{f}^{*}\right],\\ I_{c}^{*}=\frac{\left(1-\alpha \right)\beta S^{*}I_{cf}^{*}}{\alpha \left(I_{cf}^{*}+I_{f}^{*}\right)+\left(\gamma_{c}+d_{n}+d_{c}\right)-\left(1-\alpha \right)\beta S^{*}},\\ I_{cf}^{*}=\frac{\left(\alpha \beta S^{*}+\left(\alpha +\beta \right)I_{f}^{*}\right)I_{c}^{*}}{\left(d_{n}+d_{cf}+\gamma_{cf}\right)-\alpha \beta S^{*}-\alpha I_{c}^{*}-\beta I_{f}^{*}},\\ I_{f}^{*}=\frac{\left(1-\beta \right)\alpha S^{*}\left(I_{c}^{*}+I_{cf}^{*}\right)}{\beta \left(I_{cf}^{*}+I_{c}\right)+\left(\omega +d_{n}+d_{c}\right)-\left(1-\beta \right)\alpha S^{*}}. \end{array}$$

### 2.4. Basic Reproduction Number

The basic reproduction number *R*_0_ is a very important measure of the initial transmission of any infectious disease. Using the next-generation method as described by van den Driessche and Watmough [26], we have

(9) $$\begin{array}{c} F=\left[\begin{array}{ccc} \left(1-\alpha \right)\beta S^{*} & \left(1-\alpha \right)\beta S^{*} & 0\\ \alpha \beta S^{*} & \alpha \beta S^{*} & 0\\ \left(1-\beta \right)\alpha S^{*} & \left(1-\beta \right)\alpha S^{*} & \left(1-\beta \right)\alpha S^{*} \end{array}\right], \end{array}$$

(10) $$\begin{array}{c} FV^{-1}=\left[\begin{array}{ccc} \frac{\left(1-\alpha \right)\beta S^{*}}{\gamma_{c}+d_{n}+d_{c}} & \frac{\left(1-\alpha \right)\beta S^{*}}{\gamma_{cf}+d_{n}+d_{cf}} & 0\\ \frac{\alpha \beta S^{*}}{\gamma_{c}+d_{n}+d_{c}} & \frac{\alpha \beta S^{*}}{\gamma_{cf}+d_{n}+d_{cf}} & 0\\ \frac{\left(1-\beta \right)\alpha S^{*}}{\gamma_{c}+d_{n}+d_{c}} & \frac{\left(1-\beta \right)\alpha S^{*}}{\gamma_{cf}+d_{n}+d_{cf}} & \frac{\left(1-\beta \right)\alpha S^{*}}{\omega +d_{n}+d_{f}} \end{array}\right]. \end{array}$$

The basic reproduction number *R*_0_ is the largest eigenvalue of the *FV*^−1^ matrix. Now solving for the eigenvalues of *FV*^−1^ and substitute *S*^∗^ = *Λ*/*d*_*n*_ at disease-free equilibrium, we obtain

(11) $$\begin{array}{c} R_{0}=\max\left\{\frac{\left(1-\beta \right)\alpha \Lambda }{d_{n}\left(\omega +d_{n}+d_{f}\right)},\frac{\left(1-\alpha \right)\beta \Lambda }{d_{n}\left(\gamma_{c}+d_{n}+d_{c}\right)}+\frac{\alpha \beta \Lambda }{d_{n}\left(\gamma_{cf}+d_{n}+d_{cf}\right)}\right\}. \end{array}$$

Observe that

(12) $$\begin{array}{c} \frac{\left(1-\beta \right)\alpha \Lambda }{d_{n}\left(\omega +d_{n}+d_{f}\right)}=R_{0f}, \end{array}$$

is the basic reproduction number for fear epidemic,

(13) $$\begin{array}{c} \frac{\left(1-\alpha \right)\beta \Lambda }{d_{n}\left(\gamma_{c}+d_{n}+d_{c}\right)}=R_{0c}, \end{array}$$

is the basic reproduction number of coronavirus epidemic, and

(14) $$\begin{array}{c} \frac{\alpha \beta \Lambda }{d_{n}\left(\gamma_{cf}+d_{n}+d_{cf}\right)}=R_{0cf}, \end{array}$$

is the basic reproduction number of coronavirus coupled with fear epidemic.

## 3. Local Stability of the Disease-Free Equilibrium

**Theorem 1 .**

The disease-free equilibrium of the COVID-19 model (2.5) is locally asymptotically stable if *R*_0_ < 1 and unstable if *R*_0_ > 1.

**Proof**

We show that the Jacobian matrix *J*(*E*_0_) of the COVID-19 model (2.5) at *E*_0_ = (*Λ*/*d*_*n*_, 0, 0, 0) has negative eigenvalues. Further computations show that he Jacobian matrix of the COVID-19 model (2.5) at *E*_0_ is

(15) $$\begin{array}{c} J\left(E_{0}\right)=\left[\begin{array}{cccc} -d_{n} & -A & -A & -\left(1-\beta \right)\alpha S^{*}+\omega \\ 0 & B & \left(1-\alpha \right)\beta S^{*} & 0\\ 0 & \alpha \beta S^{*} & C & 0\\ 0 & \left(1-\beta \right)\alpha S^{*} & \left(1-\beta \right)\alpha S^{*} & D \end{array}\right], \end{array}$$

where *A* = (1 − *α*)*βS*^∗^ + *αβS*^∗^ + (1 − *β*)*αS*^∗^, *B* = (1 − *α*)*βS*^∗^ − (*γ*_*c*_ + *d*_*n*_ + *d*_*c*_), *C* = *αβS*^∗^ − (*γ*_*cf*_ + *d*_*n*_ + *d*_*cf*_), and *D* = (1 − *β*)*αS*^∗^ − (*ω* + *d*_*n*_ + *d*_*f*_). From the Jacobian matrix *J*(*E*_0_), we find that some of the eigenvalues are *λ*_1_ = −*d*_*n*_ and *λ*_2_ = *D* = −(*ω* + *d*_*n*_ + *d*_*f*_)[1 − (((1 − *β*)*αS*^∗^)/(*ω* + *d*_*n*_ + *d*_*f*_))]. The remaining eigenvalues are obtained from the reduced 2 × 2 matrix

(16) $$\begin{array}{c} J^{*}\left(E_{0}\right)=\left[\begin{array}{cc} B & \left(1-\alpha \right)\beta S^{*}\\ \alpha \beta S^{*} & C \end{array}\right], \end{array}$$

where *B* and *C* are as defined above.

To show that the remaining eigenvalues are negative, we need to show that the reduced Jacobian matrix *J*^∗^(*E*_0_) satisfy the Ruth-Hurwitz condition, that is, *tr*(*J*^∗^(*E*_0_)) < 0 and det(*J*^∗^(*E*_0_)) > 0. Further computations shows that

(17) $$\begin{array}{c} tr\left(J^{*}\left(E_{0}\right)\right)=B+C=-\left(\gamma_{c}+d_{n}+d_{c}\right)\left(1-\frac{\left(1-\alpha \right)\beta S^{*}}{\gamma_{c}+d_{n}+d_{c}}\right)-\left(\gamma_{cf}+d_{n}+d_{cf}\right)\left(1-\frac{\alpha \beta S^{*}}{\gamma_{cf}+d_{n}+d_{cf}}\right)<0, \end{array}$$

(18) $$\begin{array}{c} \det\left(J^{*}\left(E_{0}\right)\right)=B\times C-\alpha \beta S^{*}\left(1-\alpha \right)\beta S^{*}=1-\left[\frac{\left(1-\alpha \right)\beta \Lambda }{d_{n}\left(\gamma_{c}+d_{n}+d_{c}\right)}+\frac{\alpha \beta \Lambda }{d_{n}\left(\gamma_{cf}+d_{n}+d_{cf}\right)}\right]=\left(1-R_{0}\right)>0. \end{array}$$

Since *tr*(*J*^∗^(*E*_0_)) < 0 and det(*J*^∗^(*E*_0_)) > 0, then the proof is complete.

## 4. Global Stability of the Disease-Free Equilibrium

**Theorem 2 .**

The disease-free equilibrium is of the COVID-19 model (2.5) is globally asymptotically stable if *R*_0_ < 1 and unstable if *R*_0_ > 1.

**Proof**

To analyse the global stability of the disease-free equilibrium, we apply the Castillo-Chavez [27] approach. We write the COVID-19 model (2.5) in the form

(19) $$\begin{array}{c} \left\{\begin{array}{c} \frac{dX_{n}}{dt}=A_{1}\left(X_{n}-X_{DFE,n}\right)+A_{12}X_{e},\\ \frac{dX_{e}}{dt}=A_{2}X_{e}, \end{array}\right. \end{array}$$

where *X*_*n*_ is the vector representing the non-transmitting class and *X*_*e*_ is the vector representing the transmitting class. The disease-free equilibrium is globally asymptotically stable if *A*_1_ has negative real eigenvalues and *A*_2_ is a Metzler matrix.

From the COVID-19 model (2.5), we have *X*_*n*_ = *S* and *X*_*e*_ = (*I*_*c*_, *I*_*cf*_, *I*_*f*_)^*T*^. Further analysis gives

(20) $$\begin{array}{c} A_{1}=\left(-d_{n}\right),\\ A_{12}=\left(-a_{11}-a_{12}a_{13}\right), \end{array}$$

where *a*_11_ = *a*_12_ = (1 − *α*)*βS*^∗^ + *αβS*^∗^ + (1 − *β*)*αS*^∗^ and *a*_13_ = −(1 − *β*)*αS*^∗^ + *ω*, while

(21) $$\begin{array}{c} A_{2}=\left[\begin{array}{ccc} b_{11} & \left(1-\alpha \right)\beta S^{*} & 0\\ \alpha \beta S^{*} & b_{22} & 0\\ \left(1-\beta \right)\alpha S^{*} & \left(1-\beta \right)\alpha S^{*} & b_{33} \end{array}\right]. \end{array}$$

where *b*_11_ = (1 − *α*)*βS*^∗^ − (*γ*_*c*_ + *d*_*n*_ + *d*_*c*_), *b*_22_ = *αβS*^∗^ − (*γ*_*cf*_ + *d*_*n*_ + *d*_*cf*_), and *b*_33_ = (1 − *β*)*αS*^∗^ − (*ω* + *d*_*n*_ + *d*_*f*_).

We can clearly see that *b*_11_ = (1 − *α*)*βS*^∗^ − (*γ*_*c*_ + *d*_*n*_ + *d*_*c*_) = −(*γ*_*c*_ + *d*_*n*_ + *d*_*c*_)(1 − *R*_0*c*_), *b*_22_ = *αβS*^∗^ − (*γ*_*cf*_ + *d*_*n*_ + *d*_*cf*_) = −(*γ*_*cf*_ + *d*_*n*_ + *d*_*cf*_)(1 − *R*_0*cf*_), and *b*_33_ = (1 − *β*)*αS*^∗^ − (*ω* + *d*_*n*_ + *d*_*f*_) = −(*ω* + *d*_*n*_ + *d*_*f*_)(1 − *R*_0*f*_).

It can be easily seen that *A*_1_ has negative real eigenvalue and that matrix *A*_2_ is a Metzler matrix because all the off-diagonal elements are positive. Hence, the disease-free equilibrium *E*_0_ is globally asymptotically stable.

The existence of local stability of the disease-free equilibrium implies local stability of the endemic equilibrium. An interested individual may try to establish the global stability of the endemic equilibrium.

## 5. Impact of Fear on the Dynamics of the Model

In this section, we look into the impact of fear on the dynamics of the model. From the basic reproduction number represented by Equation (11), we have the following three cases. In case *α* = 0 and *β* > 0,

(22) $$\begin{array}{c} R_{0}=\frac{\beta \Lambda }{d_{n}\left(\gamma_{c}+d_{n}+d_{c}\right)}, \end{array}$$

which is the basic reproduction number for the classical SIR model of coronavirus fever.

In case *α* > 0 and *β* = 0, then

(23) $$\begin{array}{c} R_{0}=\frac{\alpha \Lambda }{d_{n}\left(\omega +d_{n}+d_{f}\right)}, \end{array}$$

which is the basic reproduction number for the classical SIS model of fear of contagion.

In case *α* = *β* > 0, then we expect that *d*_*c*_ = *d*_*cf*_ and *γ*_*c*_ = *γ*_*cf*_. Hence,

(24) $$\begin{array}{c} R_{0}=\max\left\{\frac{\left(1-\beta \right)\alpha \Lambda }{d_{n}\left(\omega +d_{n}+d_{f}\right)},\frac{\beta \Lambda }{d_{n}\left(\gamma_{c}+d_{n}+d_{c}\right)}\right\}. \end{array}$$

To study the variation of *R*_0*c*_,  *R*_0*cf*_, and *R*_0*f*_, with respect to *α* and *β*, we perform a 3D plot for values of *α* = [0.0 − 0.003] and *β* = []0.0 − 0.002]. The behaviour of the graphs is as shown in Figure 2. From Figure 2, we observe that *R*_0*cf*_ is between 0 and 3, while *R*_0*c*_ and *R*_0*f*_ grow as *α* and *β* increases. *R*_0*f*_ is expected to be higher than *R*_0*c*_ and *R*_0*f*_ because there are many pathways in which one can contract fear. When the disease is endemic, an individual is not expected to recovery easily from the fear of contagion; this can lead to a change in individual's behaviour and the disease prevalence.

## 6. Numerical Simulations

In this section, we carry out numerical simulation in order to study the persistence of the disease when introduced in a closed or isolated system. The initial values used in simulations are *S* = 100,  *I*_*c*_ = 1, *I*_*cf*_ = 0, *I*_*f*_ = 1, and *R* = 0. For natural death rate *d*_*n*_, we use the life expectancy of Tanzanians for the year 2019 which is 65/69 (male/female) [28]. Therefore, *d*_*n*_ = 1/65/365 = 0.000042. The time to recover from corona depends on the seriousness of the infection. Individuals presenting mild illness may recover in an average period of 2 weeks while those presenting serious or critical illness recovering in about 3 to 6 weeks [29]. For the purpose of our analysis, we use 2 weeks, and so *γ*_*c*_ = 1/14 = 0.0714. Other parameters are as indicated in Table 2.

The fear epidemic is expected to be faster than the disease epidemic because there are many ways to develop fear than are there for the coronavirus fever epidemic. An individual can develop fear from *I*_*c*_, *I*_*cf*_, or *I*_*f*_ themselves, but an individual can contract disease only by contact with *I*_*c*_ and *I*_*cf*_. Susceptible individuals self-isolate through fear as the infection of the proper disease grows. Falling of the disease incidence will cause susceptibility to return to circulation and trigger the remaining infectives to cause a second wave of infections at nearly 120 days. Figures 3(a) and 3(b) shows the variation of subpopulations for *α* < *β* and *α* > *β* using the parameter values in Table 2 except for the case where *α* > *β*. In the event that *α* > *β*, it is expected that the disease-fear death *d*_*cf*_ and the fear of contagion death rate *d*_*f*_ will increase. For the purpose of this analysis, we use *d*_*cf*_ = 0.006 and *d*_*f*_ = 0.0003 instead of the values given in Table 2.

Figure 4 shows the variation of subpopulations when *α* = *β*. In this case, we expect that *d*_*c*_ = *d*_*cf*_ and *γ*_*c*_ = *γ*_*cf*_. Here, one would expect that the disease epidemic curve and the fear epidemic curve coincide. But this is not the case actually because when fear grows, less individuals are expected to be infected.

In the event that there is no fear of contagion, that is, *α* = 0, we expect that *d*_*f*_ = 0, *ω* = 0, *d*_*cf*_ = 0, and *γ*_*cf*_ = 0. The epidemic curves for the model system are the S-curve for the SIR model of coronavirus disease as shown in Figure 5(a). On the other hand, when there is no coronavirus transmission, that is, *β* = 0, we expect that *d*_*c*_ = *d*_*cf*_ = 0 and *γ*_*c*_ = *γ*_*cf*_ = 0. The epidemic curves are the normal S-curve for the SIS fear of the contagion model as shown in Figure 5(b).

## 7. Discussion

In this paper, we used a modeling approach to investigate the dynamics of COVID-19 coupled with the fear of epidemics. To study the effect of the initial transmission of the disease, we computed the basic reproduction number *R*_0_ of the model and used to analyse the stability of the disease-free equilibrium. We also examined the effect of fear of contagion in *R*_0_ and the whole model system using numerical simulation. Analysis of the disease-free equilibrium indicates that the disease-free equilibrium of the model is locally and globally asymptotically stable when *R*_0_ < 1 and unstable otherwise. This means that the outbreak can be controlled provided that *R*_0_ < 1.

The impact of fear rate *α* and the transmission rate *β* to *R*_0_ were also examined. It was observed that increase in *R*_0_ will depend largely on the increase in *α* and *β*. Further analysis shows that as *α* and *β* increase and *R*_0*c*_ and *R*_0*f*_ grow unbounded, while *R*_0*cf*_ ranges from 0 to 3.

To analyse the variation of each subpopulation in the model with respect to time, we performed numerical simulations. The result from the numerical simulation shows that whenever there is an outbreak coupled with the fear of contagion, the disease is likely to persist in the first two months, and thereafter, it will start to slow down. As more individuals recover from fear and become susceptible, a second wave of infection is triggered in the next month. This happens in all case of *α* < *β*, *α* > *β*, and *α* = *β*.

## 8. Conclusion

COVID-19 infection will remain a potential threat to many countries globally because of its nature of transmission. Fear rate and transmission rate have been mainly seen to affect *R*_0_, which is the initial transmission of the disease. Therefore, it is essential to look into mechanisms that reduce fear and transmission simultaneously in order to reduce *R*_0_. An effective educational campaign about the nature of the disease itself and its transmission will help reduce fear among people and look for possible control mechanisms.

## Figures and Tables

**Figure 1:** Transmission diagram for the COVID-19 model.

**Figure 2:** The variation of *R*_0*c*_, *R*_0*cf*_, and *R*_0*f*_, with respect to *α* and *β*.

**Figure 3:** Time series plot for *α* < *β* and *α* > *β*.

**Figure 4:** Graphs plotted when *α* = 0.0015 = *β*, *d*_*c*_ = 0.004 = *d*_*cf*_, and  *γ*_*c*_ = 0.0714 = *γ*_*cf*_.

**Figure 5:** Time series graphs when *α* = 0 and *β* = 0.

**Table 1:** Parameters and their description.

Parameter	Description
*Λ*	Recruitment rate in human population
*d*_*n*_	Natural death rate of human
*d*_*c*_	Disease-induced death rate of human
*d*_*cf*_	Disease-and-fear-induced death rate of human
*d*_*f*_	Fear-induced death rate of human
*β*	Disease transmission rate
*α*	Disease fear rate
*γ*_*c*_	Disease recovery rate
*γ*_*cf*_	Disease and fear recovery rate
*ω*	Fear recovery rate

**Table 2:** Parameters, description, and their values.

Parameter	Description	Value (per day)	Source
*Λ*	Recruitment rate in human	1.0	Assumed
*d*_*m*_	Natural death rate of human	0.000042	[28]
*d*_*c*_	Disease-induced death rate of human	0.004	Estimated
*d*_*cf*_	Disease-and-fear-induced death rate of human	0.005	Estimated
*d*_*f*_	Fear-induced death rate of human	0.00015	Estimated
*β*	Disease transmission rate of coronavirus disease	0.0015	[29]
*α*	Fear rate of coronavirus fever	0.0010	Estimated
*γ*_*c*_	Disease recovery rate	0.0714	[29]
*γ*_*cf*_	Disease and fear recovery rate	0.0476	Estimated
*ω*	Fear recovery rate	0.010	Estimated

## Data Availability

The set of parameter values is mainly from articles similar to this work while the unavailable data especially values of parameters were estimated for the purpose of verifying results of the mathematical analysis of the model developed.
